The article "Recurrence of Early Hepatocellular Carcinoma after Surgery May Be Related to Intestinal Oxidative Stress and the Development of a Predictive Model" was retracted in 2023. Reasons: signs of a paper mill; suspected computer-generated content; unreliable results or conclusions; concerns about the data.

# Recurrence of Early Hepatocellular Carcinoma after Surgery May Be Related to Intestinal Oxidative Stress and the Development of a Predictive Model

**DOI:** 10.1155/2022/7261786

**Published:** 2022-10-04

**Authors:** Yongfei He, Tianyi Liang, Zijun Chen, Shutian Mo, Yuan Liao, Qiang Gao, Ketuan Huang, Tao Peng, Weijie Zhou, Chuangye Han

**Affiliations:** ^1^Department of Hepatobiliary Surgery, The First Affiliated Hospital of Guangxi Medical University, Nanning, Guangxi Zhuang Autonomous Region, China; ^2^Guangxi Key Laboratory of Enhanced Recovery after Surgery for Gastrointestinal Cancer, Nanning, Guangxi Zhuang Autonomous Region, China; ^3^Deputy Chief Technician of Laboratory, Baise People's Hospital, Baise, Guangxi Zhuang Autonomous Region, China

## Abstract

**Background:**

Early stage hepatocellular carcinoma (HCC) has a high recurrence rate after surgery and lacks reliable predictive tools. We explored the potential of combining enhanced CT with gut microbiome to develop a predictive model for recurrence after early HCC surgery.

**Methods:**

A total of 112 patients with early HCC who underwent hepatectomy from September 2018 to December 2020 were included in this study, and the machine learning method was divided into a training group (*N* = 71) and a test group (*N* = 41) with the observed endpoint of recurrence-free survival (RFS). Features were extracted from the arterial and portal phases of enhanced computed tomography (CT) images and gut microbiome, and features with minimum absolute contraction and selection operator regression were created, and the extracted features were scored to create a preoperative prediction model by using the multivariate Cox regression analysis with risk stratification analysis.

**Results:**

In the study cohort, the model constructed by combining radiological and gut flora features provided good predictive performance (*C* index, 0.811 (0.650-0.972)). The combined radiology and gut flora-based model constructed risk strata with high, intermediate, or low risk of recurrence and different characteristics of recurrent tumor imaging and gut flora. Recurrence of early stage hepatocellular carcinoma may be associated with oxidative stress in the intestinal flora.

**Conclusions:**

This study successfully constructs a risk model integrating enhanced CT and gut microbiome characteristics that can be used for the risk of postoperative recurrence in patients with early HCC. In addition, intestinal flora associated with HCC recurrence may be involved in oxidative stress.

## 1. Introduction

Liver cancer is a global health challenge and its incidence continues to show an increasing trend. Hepatocellular carcinoma (HCC) is the most common type of primary carcinoma of the liver, accounting for approximately 90% of all cases [1]. Cancer data show that approximately half of new HCC cases worldwide come from China each year, and HCC is the fifth most common cancer and the second leading cause of cancer death in China [2, 3]. Surgical resection is the most effective treatment modality for early-stage HCC and can significantly improve the prognosis of patients. Nevertheless, HCC still faces high recurrence rate and poor prognosis after radical resection [4–6]. Accurate prediction could aid in the development of optimal management, detection, and prevention strategies for tumor recurrence. HCC staging systems occupy a central position in prognosis and treatment [7], but none of them provide a quantifiable risk metric and are therefore insufficient to predict recurrence. Methods that can effectively predict recurrence after radical resection for early HCC are still lacking.

Imaging is an important component in the management of HCC patients. Traditional imaging modalities are based only on morphological diagnosis, discarding a large amount of information about tumor heterogeneity, which shows certain limitations in the era of emphasis on precision medicine [8, 9]. In the era of personalized treatment in oncology, radiomics can extract a large number of imaging features from imaging images and uncover highly representative quantitative histological features, which have broad clinical application prospects in guiding the diagnosis and treatment of HCC [9–12]. A study has reported that by combining radiomics, radiogenomics, and imaging techniques for the diagnosis of HCC, imaging histology can improve the accuracy of diagnosis [13]. Based on the radiomics typing of HCC, the classification rate of HCC can be improved with the addition of imaging histology features [14].In addition, improved modeling of imaging histology can predict Microvascular Invasion (MVI) and clinical survival prognosis of HCC patients [15]. However, the imaging histological features of early HCC recurrence after surgery have been poorly reported and have not been applied in the clinic.

Intestinal microecology is a complex ecosystem in which the gut microbiome and the organism interact, playing an important role in nutrient absorption, regulation of intestinal function, and immune response. Because the anatomy and physiological functions of the liver are inextricably linked to the intestine, intestinal microecology influences the development of liver disease through multiple pathways. Gut microbiome imbalance has an important relationship with the development of fatty liver disease, cirrhosis, and primary sclerosing cholangitis [16–21]. Recent studies have shown that intestinal microbes drive liver inflammatory stimuli through the “gut-liver axis” to accelerate liver carcinogenesis [22, 23].In addition, gut microbiome can influence the development and progression of hepatocellular carcinoma by regulating the expression and accumulation of immune cells [24]. Studies have demonstrated that gut microbes can be used as noninvasive diagnostic markers for liver cancer, colorectal cancer, type 2 diabetes, and cognitive impairment [25–28]. However, the potential of gut microbes as biomarkers in clinical HCC patients has not been reported.

Our aim was to construct a risk model for recurrence after early HCC based on patients undergoing hepatectomy for early HCC, extracting imaging histology and gut flora characteristics, respectively. The testing cohort was used to assess the potential of enhanced CT and gut microbiome as noninvasive biomarkers of recurrence after early HCC surgery.

## 2. Method

### 2.1. Patients

The study included 112 patients with primary early hepatocellular carcinoma who underwent radical resection in hepatobiliary surgery from September 2018 to December 2020 (Figure 1). Inclusion criteria are as follows: (1) HCC patients who were eligible for stage 0-B of BCLC staging or stage Ia-Ib of CNLC; (2) clear postoperative pathology of hepatocellular carcinoma; (3) CT plain scan of the upper abdomen and three-stage enhanced CT in the arterial, portal, and delayed stages within 1 month before surgery at our unit; (4) patients were first-time patients with no previous relevant treatment; (5) no comorbid; and (6) no antibiotics or microecological agents were used within 30 days before preoperative stool collection. Exclusion criteria are as follows: (1) CT examination was performed 1 month before surgery; (2) enhanced CT affected feature extraction due to artifacts, unsatisfactory image quality, etc.; (3) received any local or systemic antitumor therapy before surgery; (4) presence of large vessel invasion or extrahepatic metastasis, patients with BCLC stage C or above or CNCL stage IIa or above; (5) severe chronic related diseases (heart failure, systemic hypopituitarism, or autoimmune diseases); (6) previous use of drugs such as antibiotics or microecological agents within 1 month; (7) patients with other combined gastrointestinal diseases that may affect the level of gut microbiome; (8) combined with other malignancies; (9) incomplete clinicopathological data; and (10) follow-up data are not available.

### 2.2. Follow-Up

Patients were followed up after discharge according to the guidelines for the management of primary liver cancer (2019 edition) to assess postoperative recovery and recurrence. [29]. When recurrence is suspected, the diagnosis is established based on the patient's serum alpha fetal protein (AFP) and Des-gamma-carboxy prothrombin (DCP) levels, as well as abdominal ultrasonography, contrast-enhanced computed tomography (CT) or magnetic resonance imaging (MRI), and patients with confirmed recurrence of HCC receive further treatment. The follow-up deadline is February 28, 2022. Recurrence-free survival (RFS) was defined as the time from the date of surgery to the date of recurrence, metastasis, or last follow-up visit.

### 2.3. Enhanced CT Scan Equipment and Methods

CT examinations were performed using a GE 64 LightSpeed VCT and a Siemens dual-source CT scanner. A nonionic contrast agent was used for the enhancement scan (300 mgI/ml). A dollop (2.5 ml/kg) of contrast agent was injected through a forearm vein at a rate of 3 ml/s using a high-pressure syringe. Arterial (delay 22-30 seconds), venous (delay 50-55 seconds), delayed (delay 180 seconds), and continuous spiral scans (delay 6-8 seconds) were acquired at 8 mm layer thickness, 120 kV tube voltage, 280 mA beam current, and 0.5 sec/revolution. Images are stored in Digital Imaging and Communications in Medicine (DICOM) format in the Picture Archiving and Communication Systems (PACS). The extraction and analysis of radiomic features are described in the Supplementary Material.

### 2.4. Stool Sample Collection

Fresh stool samples were provided at 06:30-08:30 am after each patient's admission, divided into at least three aliquots, and stored at −80°C immediately, DNA extraction, sequencing, and data analysis are described in the Supplementary Material.

### 2.5. Model Development and Validation

We established the five Cox regression models for recurrence prediction: the OTU signature model included OTU signature only; the radiomics signature model included radiomics signature only; correspondingly, the OUT-radiomics (OR) model included OTU signature and radiomics signature; and the BCLC model and CNLC model were established based on BCLC score system and CNLC score system, respectively. All models were validated in a separate external cohort.

### 2.6. Statistical Analysis

Continuous parameters are displayed as the mean (SD) or median (IQR). Student's *t*-test and the Wilcoxon rank-sum test were then used. Categorical parameters are displayed as the number (centiles), and the Chi-squared test and Fisher's exact test were used. AFP and DC *P* values were transformed by using natural logarithm. RFS probabilities were calculated with the method of the Kaplan-Meier and compared with the log-rank test. *P* < 0.05 was statistically significant. The missing values were supplemented by mean substitution.

## 3. Result

### 3.1. Patient Characteristics

Based on the exclusion criteria, 112 HCC patients were finally eligible to the study, of whom 71 were randomly allocated to the training cohort and 41 were assigned to the testing cohort. Among the study patients, more than 90% of them were at a relatively early stage of tumor. Variables regarding to baseline clinicopathology, liver function, tumor itself, tumor stage, and surgical were well balanced between the training and testing cohort, except for the hilar occlusion time that was longer in the training cohort than that of the testing cohort (median 37.5 min vs. 31 min, *P* = 0.005). The OTU-score and the radiomic-score also had similar distributions between the training and testing cohort (Table 1).

### 3.2. Risk Factors Analysis

Univariate Cox analyses were performed in the primary cohort (Figure 2). Both OUT-score (HR[95%CI] = 1.540 [1.327−1.786], *P* < 0.001) and radiomic-score (HR[95%CI] = 5.994 [3.290−10.920], *P* < 0.001) were found to be significantly associated with RFS. Except for univariate analysis, another more 3 kinds of adjusted methods were used in the multivariate Cox analysis. The results showed that RFS was affected independently by OUT-score (Model 4: HR[95%CI] = 2.950 [2.411−3.609], *P* < 0.001) and radiomic-score (Model 4: HR[95%CI] = 5.868 [2.874−11.982], *P* < 0.001). To investigate whether the effects of OUT-score and radiomic-score can be affected by each other, we further put the two risk factors together into the Cox regression models, and we got the same results that OUT-score (Model 4: HR[95%CI] = 2.715 [2.206−3.342], *P* < 0.001) and radiomic-score (Model 4: HR[95%CI] = 6.413 [3.644−11.287], *P* < 0.001) were independent risk factors for HCC recurrence after hepatectomy (Table 2) (Supplement excel.txt 1–2).

### 3.3. Prediction Models Development and Validation

To predict RFS after hepatectomy, the five Cox regression models (OTU-score model, radiomic-score model, OTU-radiomic-score model, BCLC model, and CNLC model) were constructed in the training cohort and were validated in the testing cohort. There were no obvious violations of the proportional hazard's assumption in these five models assessed by scaled Schoenfeld residuals against time for each predictor in the radiomics models (Figure S1).

Table 3 shows that the best discriminatory ability was in the OTU-radiomic-score model with a *C* index of 0.929 (95% CI: 0.792-1.000) and 0.811 (95% CI: 0.650-0.972) in the training and testing cohorts, respectively. The prognostic performance of the OTU-radiomic-score model was showed to be superior to that of the other four predictive models in both the training and testing cohorts, demonstrating a joint effect of OTU-score and radiomic-score. Calibration plots for the OTU-radiomic-score model RFS demonstrated that the model-predicted RFS was well calibrated in both cohorts (Figure S2). When compared with the OTU-score model and the radiomic-score model, the OTU-radiomic-score model was also found to have an improved prediction ability of HCC recurrence in the time-dependent receiver operating characteristic curve analysis in both cohorts. And the prediction error curves of all models also illustrated that less prediction error was gained in the OTU-radiomic-score model (Figure 3). The integrated Brier scores for the OTU-radiomic-score model were 0.042 and 0.094 in the training cohort and the testing cohort, respectively, showing the OTU-radiomic-score model provides more precise prognostication of RFS than the other four models (Table 3). Decision curve analysis graphically demonstrated that the OTU-radiomic-score model provided larger net benefit across the range of reasonable threshold probabilities compared with the other models in both the training and testing cohorts (Figure 4). Basing on the OTU-radiomic-score model, a monogram was provided in our study (Figure 5), playing a role of convenient tool to predict the RFS of patients after hepatectomy.

### 3.4. Recurrence Risk Stratification

A prognostic index was calculated based on the OTU-radiomic-score model, with 0.22 and 3.65 as cutoff values derived from the *X*-tile analysis (Figure S3) in the whole cohort. The very model identified three risk categories of recurrence. During the follow-up, cumulative 1-year recurrence rates were 1.3%, 8.7%, and 58.3% in the low-risk, mid-risk, and high-risk group, respectively. The high-risk group and the mid-risk group were observed to have worse recurrence survival prognosis than the low-risk group (Figure 6).

### 3.5. Differentially Enriched Bacterial Taxa

To further explore the differences and potential functions between the intestinal flora of relapsed and nonrelapsed HCC, we analyzed the intestinal flora of these two groups of patients. Patients with relapsed and nonrelapsed HCC were gradually differentiated at PCA, and we further identified seven relapsed group HCC bacteria such as Ruminococcus2, Clostridium XVIII, and Fusicatenibacter and three nonrelapsed bacteria by the LEfSe analysis, which may be associated with the relapse of HCC (Figure 7) (Supplement excel.txt 3–4).

## 4. Discussion

Hepatectomy is one of the preferred treatment modalities for HCC, especially for early-stage hepatocellular carcinoma, but its 5-year postoperative recurrence rate is as high as 40%-70% [30]. Postoperative recurrence of hepatocellular carcinoma includes both intrahepatic metastasis, which is mainly due to the presence of microscopic metastases in the residual liver, and multicenter, which is due to the new tumors in the underlying cirrhotic base and underlying liver lesions [31, 32].CT, as an important noninvasive imaging modality, is an important tool for tumor diagnosis and surveillance. Quantitative imaging analysis of CT combined with machine learning allows the development of the predictive models with high accuracy and sensitivity, and imaging histology plays a key role in the diagnosis, efficacy assessment, and prediction of prognosis in HCC. In this study, we extracted preoperative CT-specific features of recurrent and recurrence-free hepatocellular carcinoma, combined with their gut microbiome characteristics, and constructed a model for the risk of recurrence after surgery for early hepatocellular carcinoma and validated it using a testing cohort, and our findings provide a reference value for the management of HCC patients.

Unlike traditional CT review, which relies on radiologists and highly qualified clinicians, imaging histology requires specialized software, reducing the demand on physicians. In addition, compared to puncture biopsy or excision of tissue for pathology, imaging histology captures a large amount of information quantitatively in a noninvasive and cost-effective manner and has good predictive power [10]. Several previous studies have reported that preoperative imaging histological features can predict early HCC recurrence [33–37], but no analysis of ROI was considered. Previous studies in breast cancer, lung cancer, and glioma have shown that tissue 5-20 mm from the tumor is strongly associated with tumor prognosis [38–40]. When surgical resection of hepatocellular carcinoma is performed, a 1 to 2 cm margin is usually recommended for hepatocellular carcinoma, and the results of the related studies have also shown that a 2 cm margin is superior to a narrow margin (<1 cm) in terms of postoperative survival [41, 42]. Looking at the site of recurrent HCC lesions, we believe it is necessary to include ROI for analysis as a way to establish a better risk model for efficacy. In this regard, we took the border of the tumor as the central point and extended it inward and outward by 5 mm to obtain more and more valuable imaging information that could help to improve the prediction of the model.

Recent animal studies have shown that the use of probiotics reduces the size of the corresponding tumors and the crosstalk between gut microbial metabolites and HCC development, while altering the levels of proinflammatory cytokines in the extraintestinal tumor microenvironment [43]. The unique portal vascular system of the liver that receives metabolites from the intestine, in addition to the presence of the enterohepatic axis of bile acids, explains to some extent the alteration of the gut microbiome that may influence the development of HCC by altering metabolites [44, 45]. Gut microbiome may vary significantly by region, nutrition, and lifestyle, with heterogeneity among organisms. However, recent studies have shown that although the gut flora differs among HCC patients in different regions, there may be universality of gut flora in HCC, suggesting the possibility of microbial markers as early screening markers [25]. These studies suggest that gut microbiome may influence the development of HCC through the gut-flora-liver axis and that gut microbiome provides new ideas for finding noninvasive biomarkers of HCC. Current research on gut microbiome focuses on markers for early diagnosis, while our study extracted characteristics and analyzed gut microbiome from early HCC patients and found that recurrence after hepatectomy in HCC patients may be related to abnormal changes in gut microbiome, and clinical interventions can be guided by early monitoring of gut microbiome changes in HCC patients, and it is also suggested that gut microbiome can be used as a predictive marker of postoperative recurrence in HCC patients.

Currently, histological studies are a common technical tool in the medical field, and histological studies contribute to accurate clinical diagnosis, personalized treatment, and monitoring of efficacy. The histological techniques allow all the molecule types in the organism to be studied, to establish databases, to screen for differentially expressed disease molecules, and to study their association with clinicopathological features. Multiparametric and modality imaging-based imaging has been widely used in the differential diagnosis of HCC, prediction of pathological outcomes, and assessment of therapeutic response [33, 46, 47]. On the other hand, gut microbes have continued to make progress in the study of HCC [48].In this study, by integrating imaging and gut microbes, we jointly screened biomarkers with good specificity, sensitivity, and noninvasiveness and successfully constructed a risk model for predicting recurrence, which provided a theoretical basis for subsequent studies. Compared to genomics, proteomics, and transcriptomics, imaging and microbiomics are more convenient and less expensive and can be more predictive while reducing patient burden.

Current studies have clarified that hepatitis B antiviral therapy is an important strategy to prevent recurrence of hepatocellular carcinoma after resection, and prophylactic immunotherapy has been reported for postoperative patients with hepatocellular carcinoma, but prophylactic hepatic artery chemoembolization is still controversial. Early identification of high-risk recurrence population is the focus and difficulty of preventing recurrence of hepatocellular carcinoma, which can identify target population for clinical trials related to antirecurrence adjuvant therapy for hepatocellular carcinoma on one hand and buy time for remedial liver transplantation on the other hand. Salvage liver transplantation can remove the tumor completely and also treat the patient's underlying liver disease to avoid the reappearance of new tumor in the residual liver, which is the best treatment option for recurrent liver cancer, but the lack of liver source severely limits the development of liver transplantation. Our model can stratify patients according to their risk factors, which helps to make individualized adjuvant treatment plans and clinical decisions at an early stage to maximize patient's life.

After hepatectomy in HCC patients, the hepatic detoxification and metabolic capacity is affected, the intestinal flora is altered, and the number of metabolites and harmful flora increases, aggravating the inflammatory reflection in the liver, aggravating the injury, and increasing the risk of recurrence. In our study, analysis of microorganisms from patients with relapsed and nonrelapsed HCC revealed that Ruminococcus2, Clostridium XVIII, and Fusicatenibacter were differentially enriched between the two and may be associated with oxidative stress. Ruminococcus is involved in the production of secondary bile acids, and its deficiency may lead to an increased intestinal inflammation and affect the host's immune system [49]. In addition, the abundance of Ruminococcus was increased by fecal microbiota transplantation (FMT), which also increased immune cells thereby enhancing antitumor immunity in mice [50]. Manganese exposure may alter the abundance of microorganisms such as Fusicatenibacter and Ruminococcus, causing an increase in lipopolysaccharide (LPS) levels, which in turn may be involved in oxidative stress [51] and neurotoxicity triggered by LPS [52, 53].

Existing studies suggest that clinicopathological parameters such as tumor load and MVI are also important in influencing the recurrence of HCC. In our study, patients were randomized, and the inclusion of clinicopathological factors in the training and testing cohorts did not improve the predictive effect of the model, so we did not include them in the subsequent analysis. Early primary hepatocellular carcinoma is not clearly defined, so we focused on patients with stage Ia-Ib of CNLC staging. Our study has some limitations. First, it is a single-center, guilt-based study with selection bias. Second, most of the cases included in the study were HCC with combined hepatitis B. Third, although all CT examinations were performed in the same unit, there was some variation in the quality of CT images. Fourth, because this study was conducted for CT combined with gut microbiome, the inclusion criteria were more stringent and the sample size was relatively small. Large samples and multicenter data are needed in subsequent studies to test its generalizability. Finally, due to lack of funding and bacterial culture conditions, we were not able to conduct more in-depth mechanistic studies.

## 5. Conclusion

In summary, this study developed a risk model to predict recurrence after early hepatectomy for hepatocellular carcinoma that combines enhanced CT features with gut microbiome. This may be useful for postoperative management of patients and personalized development of follow-up and interventions.

## Figures and Tables

**Figure 1:** Flow chart of analysis.

**Figure 2:** RFS-related risk factor analysis.

**Figure 3:** Discriminatory performance and prediction error for all models and systems in the training and testing cohorts. (a) Shows the time-related regions under the receiver operating curve (ROC) at different time points, and (b) shows the prediction error estimates for the established models and staging. Otu, operational taxonomic unit; Ra, radiomics; OR, operational taxonomic unit combines radiomics; BCLC, Barcelona clinic liver cancer; CNLC, Chinese liver cancer staging.

**Figure 4:** Decision curves for obtaining RFS using the established model and staging system in the training and testing cohorts. The *y*-axis measures the net benefit, which is calculated by adding together the benefit (true positive results) and subtracting the harm (false positive results), weighting the latter by a factor that compares the relative harm of undetected tumors to the harm of unnecessary treatment. The imaging combined with the gut microbiome model provided the best net benefit compared to the separate models and staging systems. Otu, operational taxonomic unit; Ra, radiomics; OR, operational taxonomic unit combines radiomics; BCLC, Barcelona clinic liver cancer; CNLC, Chinese liver cancer staging.

**Figure 5:** Cumulative rate of tumor recurrence for the three risk strata defined by the model.

**Figure 6:** Operational taxonomic unit combines radiomics predicted recurrence column line graph.

**Figure 7:** Differentially enriched bacterial taxa. (a) PCA showed the beta diversity evaluated by the Bray-Curtis distance between the recurrent and nonrecurrent HCC. (b) Taxonomic cladogram LEfSe showed different taxa enriched in relapsed and nonrelapsed HCC (LDA > 3, *P* < 0.05).0, non-recurrent HCC; 1, recurrent HCC.

**Table 1:** Baseline characteristics.

	Train (*N* = 71)	Test (*N* = 41)	*P* value
Gender:			0.482
Female	7 (9.86%)	2 (4.88%)	
Male	64 (90.1%)	39 (95.1%)	
Age	50.3 (9.65)	52.5 (10.3)	0.260
BMI	23.7 (3.88)	23.0 (2.71)	0.290
Child pugh:			1.000
A	70 (98.6%)	41 (100%)	
B	1 (1.41%)	0 (0.00%)	
Hepatitis_B:			0.036
Others	3 (4.23%)	7 (17.1%)	
Yes	68 (95.8%)	34 (82.9%)	
AFP	4.81 (2.64)	3.97 (2.56)	0.101
DCP	5.32 (2.47)	4.81 (2.78)	0.336
BCLC:			0.470
0	6 (8.45%)	1 (2.44%)	
A	60 (84.5%)	38 (92.7%)	
B	5 (7.04%)	2 (4.88%)	
CNLC:			0.751
Ia	38 (53.5%)	24 (58.5%)	
Ib	33 (46.5%)	17 (41.5%)	
Tumor_number:			0.264
Multiple	14 (19.7%)	4 (9.76%)	
Single	57 (80.3%)	37 (90.2%)	
Maximum_diameter	3.70 [2.50; 5.65]	3.50 [2.50; 6.00]	0.849
Tumor_location:			0.539
Left	16 (22.5%)	6 (14.6%)	
Middle	6 (8.45%)	5 (12.2%)	
Right	49 (69.0%)	30 (73.2%)	
Hilar_occlusion_time	37.5 [34.5; 55.5]	31.0 [22.0; 42.0]	0.005
Time_of_operation	245 [207; 308]	245 [215; 299]	0.878
Bleeding	200 [100; 375]	200 [100; 300]	0.831
Operation_method:			0.539
Laparoscopic	28 (39.4%)	13 (31.7%)	
Open	43 (60.6%)	28 (68.3%)	
Pathology_classification:			0.410
1&2_grade	31 (43.7%)	22 (53.7%)	
3&4_grade	40 (56.3%)	19 (46.3%)	
MVI:			0.437
No	53 (74.6%)	34 (82.9%)	
Yes	18 (25.4%)	7 (17.1%)	
Cirrhosis:			0.541
No	52 (73.2%)	27 (65.9%)	
Yes	19 (26.8%)	14 (34.1%)	
RFS	2.13 (0.91)	2.02 (0.86)	0.535
Recrudescence	0.21 (0.41)	0.24 (0.43)	0.697
Otu_score	-0.17 [-0.48; 0.32]	-0.36 [-0.48; 0.16]	0.393
Ra_score	-0.04 [-0.56; 0.48]	0.01 [-1.20; 0.52]	0.548

**Table 2:** Evaluation relationship between radiomic-score and OTU-score and HCC recurrence in the Cox proportional hazards models.

	Model 1 (*P*, HR[95% CI])	Model 2 (*P*, HR[95% CI])	Model 3 (*P*, HR[95% CI])	Model 4 (*P*, HR[95% CI])
Radiomic-score	<0.001, 5.994[3.290-10.920]	<0.001, 5.856[3.159-10.858]	<0.001, 5.284[2.776-10.059]	<0.001, 5.868[2.874-11.982]
Radiomic-score^∗^	<0.001, 5.416[3.021-9.710]	<0.001, 5.343[2.955-9.659]	<0.001, 4.360[2.455-7.744]	<0.001, 6.413[3.644-11.287]
OTU-score	<0.001, 1.540[1.327-1.786]	<0.001, 1.533[1.321-1.780]	<0.001, 2.881[2.357-3.521]	<0.001, 2.950[2.411-3.609]
OTU-score^∗^	<0.001, 1.348[1.140-1.593]	<0.001, 1.357[1.146-1.607]	<0.001, 2.163[1.763-2.655]	<0.001, 2.715[2.206-3.342]

Note: Model 1: we did not adjust any other parameter; Model 2: we constructed a minor adjusted model, which is adjusted for gender and age; Model 3: we adjusted the model for clinical important parameters, adjusting for gender, age, Child-pugh grade, AFP, DCP, tumor number, tumor maximum diameter, blood loss, pathology classification, MVI, and liver cirrhosis; Model 4: in this model, we adjusted for all parameters except for parameters that have existing collinearity, adjusting for gender, age, BMI, Child-pugh grade, hepatitis, AFP, DCP, tumor number, tumor maximum diameter, tumor location, hilar occlusion time, blood loss, pathology classification, MVI, and cirrhosis; ^∗^: we added radiomic-score and OTU-score as an adjusting factor into each of these models and further explore the relationship between radiomic-score and HCC recurrence; HCC, hepatocellular carcinomar.

**Table 3:** Prognostic performance of radiomics combined with the gut microbiome models compared with staging systems.

	Train				Test			
Models	*C* index	Time-dependent AUC	IBS	*P* value	*C* index	Time-dependent AUC	IBS	*P* value
OTU	0.824 (0.729-0.919)	0.848	0.077	0.032	0.751 (0.557-0.945)	0.753	0.092	0.268
Ra	0.847 (0.726-0.968)	0.895	0.059	0.033	0.791 (0.619-0.962)	0.840	0.097	0.111
OR	0.900 (0.792-1.000)	0.929	0.042	Ref	0.811 (0.650-0.972)	0.859	0.094	Ref
BCLC	0.612 (0.379-0.845)	0.500	0.114	0.013	0.615 (0.097-1.000)	0.500	0.138	0.233
CNLC	0.598 (0.339-0.858)	0.569	0.114	0.013	0.769 (0.481-1.000)	0.652	0.132	0.373

Otu, operational taxonomic unit. Ra, radiomics. OR, operational taxonomic unit combines radiomics. BCLC, Barcelona clinic liver cancer. CNLC, Chinese liver cancer staging.

## Data Availability

Data are available from the author upon reasonable requests.

## Supplementary Materials

Supplementary Materials Figure-S1: proportional risk. Figure-S2: correction curve. Figure-S3: *X*-tile analysis. Supplementary material, Intestinal microbiota characteristics and CT feature extraction method. Supplement excel.txt 1; genus abundance. Supplement excel.txt 2; genus count. Supplement excel.txt 3; PCA value. Supplement excel.txt 4; LEfSe.
